# The Consequences of COVID-19 on Breast Cancer Screenings in an Underserved Urban Population and the Screening Access of Value for Essex Program’s Efforts to Control the Damage

This article has been retracted.

**DOI:** 10.7759/cureus.42338

**Published:** 2023-07-23

**Authors:** William J Lee, Yash Shah, Nidhi Patel, Albert Ku, Anibian Rodriguez, Magdalena Salvador

**Affiliations:** 1 Radiology, Rutgers University New Jersey Medical School, Newark, USA; 2 Radiology, Drexel University College of Medicine, Philadelphia, USA

**Keywords:** radiology oncology, breast cancer screening barriers, screening mammogram, covid 19, underserved populations

## Abstract

Objective: This study aims to examine the impact of the COVID-19 pandemic on breast cancer screening in an underserved population, identify patient barriers, and discuss strategies to promote the importance of screening.

Methods/operations: The Rutgers New Jersey Medical School Screening Access of Value for Essex (SAVE) program delivers cancer prevention services to the most vulnerable population in Essex County, New Jersey. The SAVE program was shut down from March 2020 to June 2020 due to COVID-19. The number of mammograms performed 18 months before the pandemic (September 2018 to March 2020) and 18 months after the shutdown of the program (July 2020 to December 2021) were recorded. A calling project was created in response to the pandemic to educate patients about COVID-19 precautions and provide healthcare and social services resources.

Results: There was a 15.4% reduction in screening mammograms during the post-shutdown period (1,459 pre-COVID-19 versus 1,234 post-shutdown). The number of diagnostic mammograms increased from 264 to 272. The calling project spoke with 1,548 patients and identified the following concerns: exposure to COVID-19, language barriers, and lack of health insurance.

Conclusion: Although COVID-19 had a profound impact on most patients, especially in the realm of breast cancer screening, the implementation of the SAVE program's strategies such as transitioning to an appointment-only system has helped minimize the negative impacts. Reaching out to the patients, partnering with community organizations, and promoting SAVE services have played a vital role in encouraging more patients to have screening done.

## Introduction

During the peak of the COVID-19 pandemic, all patients had a substantially harder time accessing various modalities of healthcare including annual follow-ups, elective procedures, screening exams, and other routine health services [1,2]. The fear of contracting COVID-19 coupled with state-mandated lockdowns meant that very few individuals were leaving their homes, let alone seeing their physicians. In an attempt to react to the ongoing pandemic, national health organizations such as the Centers for Medicare & Medicaid Services issued recommendations to postpone screening and preventive visits for the time being in an effort to control the spread of COVID-19 [3]. Retrospective national analyses that aimed to quantify the overall decrease in the number of screening exams report that the number of screening mammograms completed during the peak of the pandemic in April 2020 was only 3.7% of the monthly average before the outbreak of COVID-19 [4].

All the barriers that prevented patients from accessing healthcare during the COVID-19 pandemic were magnified in underserved urban populations where a majority of residents require additional services such as public transportation, language interpreter services, and assistance-based payment programs [5]. Due to government shutdowns, these key services that are essential for ensuring vulnerable populations receive high-quality care were not available. As it stands, racial and ethnic minority groups such as Blacks and Hispanics have been shown to have higher incidences of disease and poorer health outcomes irrespective of the COVID-19 pandemic [6]. Black women in particular have been shown to have higher morbidity and mortality rates from breast cancer [7].

It is especially important to acknowledge that this detrimental phenomenon is exacerbated in places such as Essex County, which house large populations of historically underserved communities due to longstanding barriers to healthcare that have persisted for years on end. Essex County is one of New Jersey’s most vulnerable patient populations with a demographic composed of over 60% of residents who identify as either Black or Hispanic [8]. This patient population is not only underserved but was also severely affected by the pandemic. Prior to the COVID-19 pandemic, there were several community-health programs that existed to provide patients in Essex County with a wide variety of health-related services. One of these programs is called the Rutgers New Jersey Medical School Screening Access of Value for Essex (SAVE) program, which is one of the oldest funded New Jersey Cancer Education and Early Detection (NJCEED) programs. The SAVE program delivers cancer prevention services such as breast exams, screening mammograms, pap smear testing, and much more to the most vulnerable population in Essex County. These screening exams are offered at no cost to women who meet all of the NJCEED criteria, such as being between 21-64 years old currently, being New Jersey residents, having no insurance, and having an income at or below 250% of the federal poverty line [9].

The SAVE program was shut down from March 2020 to June 2020, which ultimately meant that patients were unable to obtain many essential preventive health services. To combat the potential harms of the pandemic on breast screenings, the SAVE program developed a calling project to educate patients about COVID-19 precautions and provide healthcare and social services resources. Strategies to minimize COVID-19 exposure such as wearing masks, social distancing, and proper hand hygiene were provided to patients prior to screening visits via phone. Lists of social service resources such as locations of outdoor “Fresh Produce Pop Up Markets” were created and distributed to patients especially those who were concerned about COVID-19 exposure from grocery stores. The objective of this study is to determine how breast cancer screenings were impacted in the underserved population of Essex County due to the COVID-19 pandemic.

This article was previously presented in the form of an electronic poster presentation at the 2022 American College of Radiology Annual Meeting on April 24, 2022.

## Materials and methods

Pre-COVID-19 operations

The SAVE program is the only NJCEED screening program that operates in Essex County, New Jersey. This is the only health screening program in Essex County, which provides free breast and cervical cancer screenings for residents and has a primary focus on targeting the underserved population in this county. Traditionally, SAVE operates as a community outreach model. This is accomplished through the use of a mobile mammography van (Figure 1) and more than 55 community partners that include various health departments, churches, and other community organizations throughout Essex County (Figure 2). Operating at least three times a week, the mobile mammography van travels to the various outreach sites to ensure that the health screenings are accessible to patients that do not have transportation. At each screening site, 15-20 patients that meet NJCEED criteria are scheduled per screening site on a first-come-first-serve basis. At each appointment, patients receive cancer education as well as breast and cervical cancer screenings.

**Figure 1:** Mobile mammography van used for breast and cervical screenings (the top image shows the exterior and the bottom image shows the interior)

**Figure 2:** Map of SAVE screening sites SAVE: Screening Access of Value for Essex.

Post-COVID-19 operations

To minimize contact and stop the spread of COVID-19, the traditional first-come-first-serve basis was transitioned to an appointment-only system. This was done to allow for adequate time between each appointment to reduce potential exposure from one patient to the next and to maximize social distancing. In a similar light, patient information and cancer education were provided via phone prior to the appointment to reduce the amount of time each patient would physically take in person.

Calling project

In response to the COVID-19 pandemic, a calling project was developed to provide COVID-19 precautions and receive direct feedback from our active and newly scheduled patients. Patients were reached via phone call and were provided different strategies to protect themselves from contracting COVID-19 including social distancing, wearing masks, and resources for COVID-19 testing. Patients were able to voice on the phone about the obstacles they currently faced to acquiring their breast and cervical screening services, which were obtained prior to appointments, and these verbal responses from patients were recorded.

Metrics

The 18 months prior to the shutdown of the SAVE program from September 2018 to March 2020 were defined as the pre-COVID-19 time period, and the 18 months following the restart of the SAVE program after its shutdown from July 2020 to December 2021 were defined as the post-COVID-19 time period. The total number of screening mammograms and diagnostic mammograms were recorded for both the pre-COVID-19 and the post-COVID-19 time periods. Pre- and post-COVID-19 shutdown era screening and diagnostic mammograms were compared via Chi-squared tests. All analyses and descriptive statistics were conducted using Microsoft Excel (Microsoft Corporation, Redmond, Washington). To assess the progress of the calling project, the total number of patients that were contacted as well as the major concerns each patient had on accessing their screening services were recorded.

## Results

A 15.4% reduction in screening mammograms occurred subsequent to the shutdowns demarcating the post-COVID-19 period (1,459 pre-COVID-19 shutdown versus 1,234 post-COVID-19 shutdown). Tangential to this reduction in screening mammograms, the number of diagnostic mammograms performed increased by 3% (264 pre-COVID-19 shutdown versus 272 post-COVID-19 shutdown).

Subsequent Chi-squared tests sought to evaluate the differences between screening and diagnostic mammograms with respect to the pre- and post-COVID-19 shutdown time frame. Chi-squared analysis for the number of screening mammograms conducted pre-COVID-19 shutdown when compared to post-COVID-19 shutdown yielded a p-value of less than 0.001, while analysis for the number of diagnostic mammograms conducted in the same study time frame yielded a p-value of 0.0622 (Table 1).

**Table 1:** Statistical analysis of pre- versus post-COVID-19 screening and diagnostic mammograms

Pre- versus post-COVID-19 screening and diagnostic mammograms		
Chi-squared test		
Pre- vs. post-COVID-19 screening mammograms	Pre: 1,459 vs. post: 1,234	p < 0.001
Pre- vs. post-COVID-19 diagnostic mammograms	Pre: 264 vs. post: 272	p = 0.622
Descriptive statistics		
Percent change of screening mammograms in pre- vs. post-COVID-19 shutdown era		-15.40%
Percent change of diagnostic mammograms in pre- vs. post-COVID-19 shutdown era		3.00%
Proportion of COVID-19 shutdown era screening mammograms conducted pre-COVID-19 shutdown		54.20%
Proportion of COVID-19 shutdown era diagnostic mammograms conducted pre-COVID-19 shutdown		49.30%

Looking at the pre- and post-COVID-19 shutdown era in conjunction, it was found that 54.2% of screening mammograms were conducted pre-shutdown, and 49.3% of diagnostic mammograms were conducted post-shutdown.

The calling project spoke with 1,548 patients during the post-COVID-19 shutdown period and identified the most prevalent and recurrent themes among patient concerns: exposure to COVID-19, language barrier, and lack of health insurance. All the concerns that were most consistently vocalized by patients had a connection to the aforementioned themes. Subsequent measures taken by the project to combat these issues included the following parameters: education regarding hospital procedures implemented to limit COVID-19 exposure and reassurance to patients in their own language with the use of language interpreter services. Language interpreters for Spanish, Portuguese, Haitian Creole, and French Creole were used. Flyers were created and distributed to patients to promote SAVE services and the development of best practice plans to keep patients safe, such as social distancing, hand hygiene, and the use of masks.

## Discussion

The study ultimately observed a 15.4% reduction in screening mammograms during the post-COVID-19 shutdown period. This is extremely problematic given its context within an increase in screening eligibility resulting from the pandemic. The study observed a complex interplay between the increases and decreases in screening mammogram demand due to the pandemic’s effect on already existing systemic factors such as insurance coverage, access to transportation, and language barriers. The Chi-squared analysis comparing the number of screening mammograms conducted pre- and post-COVID-19 shutdown demonstrated a statistically significant difference between these two time frames while demonstrating no statistically significant difference in diagnostic mammograms. While there is no single factor that clearly led to the observed increase in the number of diagnostic mammograms in the post-COVID-19 shutdown period, one of the most likely explanations is an accumulation of diagnostic screening mammograms that were previously scheduled. The previously scheduled appointments would have been rescheduled to a later date due to the COVID-19 shutdown. The total of these rescheduled appointments in addition to the new diagnostic mammograms that were ordered during the post-COVID-19 shutdown period would ultimately lead to an increase in the observed number of diagnostic mammograms. This observed increase in diagnostic mammograms also represents the success of the SAVE program in matching the increased demand for diagnostic mammograms.

Due to the COVID-19 pandemic, there was an overwhelming increase in unemployment, which subsequently resulted in many individuals losing the insurance plan provided to them by their job [10]. This was then followed by a resulting increase in the number of NJCEED-eligible residents. Small Area Health Insurance (SAHIE) estimated that in 2017, 11.5% were uninsured in Essex County. However, in 2020, this estimate had increased from 0.9% to 12.4% in the county [11,12]. Therefore, as a result of the COVID-19 shutdown period, more patients were now eligible to receive a screening mammogram under the NJCEED eligibility guidelines. This means that the 15.4% reduction in screening mammograms underestimates the severity of the resulting decrease in screenings in the scope of an increased eligible patient pool.

Despite the aforementioned causes for increasing screening eligibility, there were also a few considerable factors causing a decrease in screening demand. Marginalized communities have a longstanding history of public distrust toward the healthcare system, and this is a very significant obstacle in Essex County, which houses a large number of historically underserved and marginalized communities [13]. Historical occurrences of repeated acts of systemic bias, racism, and decreased quality of care have led to an overall sense of distrust within these communities of Essex County [14]. This was further propagated through the COVID-19 pandemic, which introduced another obstacle to accessing care through the forms of misinformation and uncertainties that ran rampant during the beginning of the pandemic [15]. Each individual’s perception of the threat from the COVID-19 virus became another obstacle to seeking routine screening mammograms.

The SAVE program quickly adopted a two-pronged approach consisting of patient education regarding COVID-19 best practices and identifying patient concerns to minimize the decrease in screenings, all accomplished through the implementation of the calling project. The program quickly understood the role that COVID-19 played on the already existing barriers to care for the underserved community within Essex County, and the goal of the project was to prioritize educational initiatives to reduce the impact of COVID-19 on these at-risk communities. The program simultaneously was able to start assessing the major concerns that alienated these patients from the healthcare system during the post-COVID-19 shutdown period. These included concerns about exposure to COVID-19, language barriers, and lack of health insurance.

The current study parallels others in finding that the COVID-19 pandemic was a very strong determinant of the decrease in screening mammograms over the past few years. It is therefore imperative that other groups, institutions, and organizations follow the example set forth by the SAVE program and the calling project to do all that they can to alleviate the disproportionate decrease in screening mammograms that these specific communities were afflicted with during the peak period of the pandemic. There needs to be a replication of the two-pronged approach employed by the SAVE program, which not only sought to provide screenings to marginalized communities but also sought to communicate with them regarding their unique concerns, obstacles, and challenges to promote community-based education for long-lasting change and impact.

While this is the first study to assess how the Essex County community was impacted by the COVID-19 pandemic in regard to breast cancer screening, the major limitation of this study was the confinement of the pre- and post-shutdown periods to only 18 months. Defining longer shutdown periods would have allowed for the evaluation of more distinct longitudinal trends in breast cancer screenings and ultimately would have provided a more definitive answer to how the number of screening and diagnostic mammograms changed. An additional limitation includes restricted demographic data collection. Collection of the patient’s race and ethnicity would allow for the analysis of individual demographic groups to assess if changes in breast screening cancer screening were more prominent in particular demographics. Marginalized communities are typically composed of minority groups that have been shown to have higher distrust of the healthcare system as mentioned earlier. This would allow for more targeted action plans like more community outreach and patient education toward these specific groups to address the causes of screening deficiencies.

## Conclusions

The COVID-19 pandemic negatively impacted the most vulnerable patients in Essex County, New Jersey, in regard to breast cancer screenings. The reduction in screening mammograms can be attributed to multiple factors including fear of illness, lack of transportation, lack of insurance, and other barriers to healthcare. The SAVE program is the only NJCEED screening program that operates in Essex County, New Jersey, and has a mission of providing healthcare services to the underserved community in this county. To mitigate the consequences of the COVID-19 pandemic and government shutdown, the SAVE program implemented a calling project to promote SAVE services to ensure that patients can safely access their screening services while minimizing risks. The success of the program can be demonstrated by the statistically insignificant difference in diagnostic mammograms before and after the COVID-19 shutdown (p = 0.622). However, the decrease in screening mammograms represents a similar trend that is observed in previous literature regarding COVID-19 and breast cancer screening nationwide. Expansion of SAVE services with additional community sites and more available appointments will be necessary to accommodate additional patients, especially with future emerging infectious diseases.
